# Active Ingredients and Potential Mechanisms of the Gan Jiang-Huang Qin-Huang Lian-Ren Shen Decoction against Ulcerative Colitis: A Network Pharmacology and Molecular Docking-Based Study

**DOI:** 10.1155/2021/1925718

**Published:** 2021-09-08

**Authors:** Ce Zhou, Hang Zhou, Furong Zhang, Liangliang Hao, Jing Guo

**Affiliations:** ^1^Department of Proctology, Hospital of Chengdu University of Traditional Chinese Medicine, Chengdu 610072, China; ^2^School of Basic Medical Sciences, Chengdu University of Traditional Chinese Medicine, Chengdu 610072, China; ^3^College of Health Preservation and Rehabilitation, Chengdu University of Traditional Chinese Medicine, Chengdu 610072, China; ^4^School of Clinical Medicine, Hospital of Chengdu University of Traditional Chinese Medicine, Chengdu 610072, China

## Abstract

**Background:**

Ulcerative colitis (UC), a chronic and nonspecific inflammatory bowel disease, seriously affects the quality of patients' life. Han Re Bing Yong Fa (treating diseases with both cool- and warm-natured herbs) is a classical therapeutic principle of traditional Chinese medicine (TCM), which is often used to treat chronic diseases, including UC. The Gan Jiang-Huang Qin-Huang Lian-Ren Shen decoction (GJHQHLRSD), a representative of Han Re Bing Yong Fa, is effective in alleviating inflammatory symptoms in UC. However, the pharmacological mechanism underlying its anti-inflammatory effect remains unclear.

**Methods:**

A network pharmacology strategy, including the construction and analysis of the drug–disease network, was used to explore the complex mechanism of GJHQHLRSD treatment of UC. In addition, molecular docking technology was used to preliminarily examine the binding ability of the potential active components and core therapeutic targets of GJHQHLRSD.

**Results:**

The network pharmacology results revealed 140 targets of GJHQHLRSD which are involved in UC. The PPI network analysis identified seven target genes: *BCL2L1, NR3C1, ALOX5, S1PR5, NR1I2, CYP2D6*, and *LPAR6.* The molecular docking results revealed that the following displayed strongest combined effects: *EGFR* with kaempferol, *ERK1* with worenine, *STAT3* with Palmidin A, *BCL2L1* with diop and *VEGFA* with ginsenoside Rg3. The KEGG and gene ontology enrichment analyses results indicated that GJHQHLRSD functions by regulating the EGFR signaling pathway in UC treatment. Other effective biological processes involved in UC treatment included cancer-related as well as inflammation and viral infection signaling pathways, such as the “MicroRNAs in cancer,” “TNF signaling pathway,” and “JAK-STAT signaling pathway.”

**Conclusions:**

This study reflects the multicomponent, multitarget, and multipathway characteristics of the action mechanism of GJHQHLRSD in treating UC. Furthermore, it helps better understand the TCM therapeutic principle of Han Re Bing Yong Fa and explore novel candidate drug targets for UC treatment.

## 1. Introduction

Ulcerative colitis (UC), a chronic, relapsing, and nonspecific inflammatory disease, affects several million individuals worldwide. UC is an inflammatory bowel disease (IBD), and its aetiology and pathogenesis are not yet fully understood. Currently, it is believed that IBD is a complex genetic disease that is instigated and amplified by the confluence of multiple genetic and environmental variables that perturb the immune–microbiome axis [1]. However, drug resistance, dependence, and adverse reactions have further limited the clinical efficacy. The prevalence of UC is increasing globally, but the clinical benefits of current treatments are controversial [2]. With a long-term ineffective treatment, UC is likely to develop into colon cancer, and up to 15% of patients may need surgical resection of the colon during later stages of the disease [3]. Hence, patients with colitis-associated cancer (CAC) suffer from more severe pain and struggle with economic burden. UC is now becoming a complex problem for physicians worldwide owing to the lack of effective treatments.

Traditional Chinese medicine (TCM) plays an important role in China's public health system, particularly in the treatment and management of chronic diseases such as UC. Currently, studies have been focusing on TCM as an alternative therapy for UC; however, there are some limitations in terms of TCM use in clinical practice, such as the lack of full guidance from the theoretical basis of TCM and the use of complex and multiflavoured herbs which are not used frequently in clinical practice. For instance, the TCM formula Guchang Zhixie Wan (GCZXW) exerts a protective effect on IBD through the STAT3/NF-kB/IL-6 pathway, and the active ingredients of the Banxia Xiexin decoction (BXXXD) primarily act on IL-4, IL-10, IL-1*β*, and TNF-*α* [4, 5]. However, several types of herbs are used in GCZXW, which hinders further study. Furthermore, BXXXD is frequently used in gastritis treatment but seldom used in UC treatment. TCM focuses on syndrome differentiation and treatment because different patients present with different syndromes. Han Re Bing Yong Fa (treating diseases with both cool- and warm-natured herbs) is a classical therapeutic principle of TCM, which is often used to treat diseases involving complex pathogenesis. Han Re Bing Yong Fa can enhance the curative effect by guiding the compatibility of one or more cold herbs with warm herbs. The *Gegen Qinlian* decoction (GGQLD), *Wumei* pill (WMP), *Shaoyao* decoction (SYD), and Gan Jiang-Huang Qin-Huang Lian-Ren Shen decoction (GJHQHLRSD) apply this principle and are representative prescriptions for UC treatment. The efficacy of GGQLD, WMP, and SYD has been demonstrated in several pharmacological and animal studies, which showed that formulas based on Han Re Bing Yong Fa can improve intestinal barrier function, alleviate UC, and delay cancer development [6–10]. However, to our knowledge, no studies have explored the mechanism and active components of GJHQHLRSD for UC treatment.

In China, GJHQHLRSD is primarily used to treat patients with gastrointestinal diseases, especially those with large intestinal damp-heat syndromes, which lie in the indication scope of Han Re Bing Yong Fa. GJHQHLRSD comprises Gan Jiang (Zingiberis Rhizoma), Huang Qin (Radix Scutellariae), Huang Lian (Coptidis Rhizoma), and Ren Shen (Ginseng Radix et Rhizoma). The Zingiberis Rhizoma decoction has been found to reduce colitis in mice by reducing the expression levels of TNF-*α*, IL-1*β*, IL-6, and IL-10 [11]. The respective active components of Radix Scutellariae and Coptidis Rhizoma can improve intestinal barrier function, thus alleviating the adverse symptoms in patients with UC [12, 13]. Moreover, the Huang Lian-Jiedu decoction has been demonstrated to alleviate UC in mice by regulating the metabolism of arachidonic acid and glycerophospholipid and may evolve into a new antiulcer drug in the future [14]. UC is caused by various genetic and environmental factors; therefore, it was hypothesized that the treatment needs a combination of multitarget drugs, similar to AIDS cocktail therapy. The current research on TCM in the treatment of UC reflects the advantages of a multitarget and multichannel approach. The current literature presents network pharmacology studies on a single herb among those included in this prescription; however, no comprehensive study has focused on the formula as a whole. A network pharmacology-based research is needed for understanding the mechanism of GJHQHLRSD in UC treatment. Therefore, this study aimed to help better understand the Han Re Bing Yong Fa therapeutic principle, clarify the possible mechanism of GJHQHLRSD in UC treatment, and explore novel candidate drug targets for UC treatment based on network pharmacology analysis results to provide a reference for future confirmatory studies.

## 2. Materials and Methods

### 2.1. Effective Chemical Composition and Targets of GJHQHLRSD

Data on the active compounds and protein targets of four herbs were retrieved from the Traditional Chinese Medicine Systems Pharmacology Database and Analysis Platform (TCMSP, https://lsp.nwu.edu.cn/tcmsp.php). The drug feasibility was evaluated by oral bioavailability (OB) and drug likeness (DL) indices. In this study, molecules with OB of ≥30% and DL of ≥0.18 were considered active compounds. The structures of GJHQHLRSD components were obtained from the PubChem database (https://pubchem.ncbi.nlm.nih.gov/) and were imported into the Swiss target prediction database (STP, https://www.swisstargetprediction.ch/); targets with a prediction score of >0 were considered the drug targets. The databases and tools were last accessed on 13 February, 2021.

### 2.2. Potential Disease Target Genes

Potential disease targets associated with UC were collected from the OMIM (https://omim.org/), DisGeNET (https://www.disgenet.org/), and GeneCards (https://www.genecards.org/) databases. The GeneCards database establishes the correlation ranking between genes and diseases and provides the gifts and score algorithm [15]. The common targets of drugs and diseases are obtained by intersecting GJHQHLRSD component targets with disease targets. Through the software analysis and screening, the overlapping genes between active drug compounds and diseases were depicted using Venn diagram (https://bioinformatics.psb.ugent.be/webtools/Venn/). Finally, Cytoscape software (Version 3.7.1) was used to map the disease network of drug components.

### 2.3. Construction of the Protein-Protein Interaction Network and Key Gene Screening

The identified overlapping target genes were introduced into the STRING network platform (https://string-db.org/). “*Homo sapiens*” was chosen, and a confidence score of >0.9 was set to predict the interactions. The protein-protein interaction (PPI) network analysis results were saved in TSV format and imported into Cytoscape software (https://www.cytoscape.org/). Key genes were screened using the CytoHubba module and MCODE plug-ins [16]. First, the MMC algorithm of CytoHubba plug-in was used to calculate the gene core degree; the genes with the top seven MMC scores were selected. Next, the MCODE plug-in was applied to set the K-core to 2 and obtain the intersection of the three core modules by clustering. Moreover, the identified genes considered the key genes involved in GJHQHLRSD treatment for UC.

### 2.4. Gene Ontology and Kyoto Encyclopedia of Genes and Genomes Pathway Enrichment Analysis

Gene ontology (GO) analysis was performed using the WebGestalt online tool (https://www.web-gestalt.org/) [17]. The Go enrichment analysis included the biological process (BP), cellular component (CC), and molecular function (MF). The results showed that the GO function with an FDR value of <0.05 indicated significant enrichment. The Kyoto Encyclopedia of Genes and Genomes (KEGG) database (https://www.genome.jp/kegg/) was used for the systematic analysis of molecular networks with interacting genes. To assess a possible mechanism of GJHQHLRSD in treating UC, the KEGG pathway enrichment analysis was performed via DAVID Bioinformatics Resources (https://david.ncifcrf.gov). Top 20 significant pathway items were considered important and were presented via a bubble graph. The abovementioned database was last accessed on 14 February, 2021.

### 2.5. Molecular Docking Analysis

First, the SDF formats of small ligand molecules were downloaded from the PubChem database and then converted to the PDB format using the Open Babel software (version 3.0.0). Second, the PyMOL software (version 2.3.6) was used to remove water molecules; the original ligand was isolated from the core target protein. The processed protein targets were imported into the AutoDock software (version 4.2.0) for hydrogenation, the total charge was calculated, the atomic type was set, and the file was saved in PDBQT format. Finally, the mol2 structures of the corresponding part of the core targets were downloaded from the TCMSP database and saved in PDBQT format. The AutoDock-Vina software (version 1.1.2) was used to perform molecular docking and comprehensively scored the receptor-ligand complex to evaluate its affinity.

The flowchart of the network pharmacology approach used in this study is shown in Figure 1.

## 3. Results

### 3.1. Identification of GJHQHLRSD Compounds

The active components of Zingiberis Rhizoma, Radix Scutellariae, Coptidis Rhizoma, and Ginseng Radix et Rhizoma were identified using the TCMSP database, and 75 potential active components were obtained. A total of 836 drug targets were selected by retrieving GJHQHLRSD from the STP database. The keyword “ulcerative colitis” was searched in the OMIM, DisGeNET, and GeneCards databases, and 906 disease targets were obtained after deduplication. Finally, the intersection images of GJHQHLRSD-UC targets were created using the Venny 2.1 online software. After mapping the UC-related genes with the targets of active compounds, 140 intersected genes were identified (Figure 2).

### 3.2. Topological Network Analysis

Four active components were deleted owing to a lack of intersection with the disease target, thus obtaining 71 active components. Data of 71 active components and 140 overlapping target genes were entered into the Cytoscape software for creating network diagram. The isolated components were deleted because of the lack of intersection with the targets, and then, a network diagram of the interaction between the drug component and target disease was drawn (Figure 3). A network analyzer was used to perform a topology analysis on the network graph, wherein the degree value represented the number of associations between the component and the target. The greater the degree value of the target point, the more important is its component.

### 3.3. PPI Network and Key Gene Analysis

The PPI network was obtained from the STRING database and visualized using the Cytoscape software. The minimum confidence was set to 0.40 to construct the PPI network and hide independent target protein nodes. The PPI network nodes represent the proteins, and the edges represent the interactions between the proteins. The importance and priority of proteins were analyzed based on network results, and seven target genes were obtained (Figure 4). The seven core genes were related to cell apoptosis (B cell lymphoma-2 like 1 (*BCL2L1*)), sphingosine-1-phosphate receptor 5 (*S1PR5*)), inflammation (arachidonate 5-lipoxygenase (*ALOX5*)), hormones (nuclear receptor subfamily 3 group C member 1 (*NR3C1*)), nuclear receptor subfamily 1 group I member 2 (*NR1I2*)), a monooxygenase gene with a detoxification effect (cytochrome P450 subfamily IID 6 (*CYP2D6*)), and a cell signal transduction gene with immune regulation (lysophosphatidic acid receptor 6 (*LPAR6*)).

### 3.4. GO Enrichment Analysis

After searching the 140 common targets in the R language software, BP, CC, and MF were selected for the GO analysis. The GO results showed that the intersection genes included multiple biological processes. The effect of GJHQHLRSD on UC is a result of complex multichannel synergy. In addition, the GO enrichment analysis was performed for top 20 BPs (Figures 5(a) and 5(b)). On the basis of the enrichment results, three most remarkable BPs were positive response regulation to external stimulus (GO:0032103), molecule of bacterial origin (GO:0002237), and lipopolysaccharide (GO:0032496). The MCODE algorithm was used to identify the mechanism underlying the positive regulation of the responses to external stimuli, molecules of bacterial origin, and lipopolysaccharides. The genes involved in these BPs are shown in Figures 5(c)–5(e)).

### 3.5. KEGG Enrichment Analysis

Data of a total of 140 potential targets of GJHQHLRSD for UC were uploaded to the DAVID database for the enrichment analysis, and 141 pathways with a *P* value of <0.05 were obtained. The results of top 20 pathways were visualized as a bubble diagram (Figure 6), which suggested that GJHQHLRSD treatment of UC is related to the tyrosine kinase inhibitor resistance of the epidermal growth factor receptor (EGFR). In addition, the analysis results included cancer-related as well as inflammation and virus infection signaling pathways, such as the “MicroRNAs in cancer,” “TNF signaling pathway,” and “JAK-STAT signaling pathway.”

### 3.6. Molecular Docking Analysis

The top five target genes were selected, including *BCL2L1*, *EGFR*, extracellular regulated kinase 1 (*ERK1*), signal transducer and activator of transcription 3 (*STAT3*), and vascular endothelial growth factor A (*VEGFA*), which play a significant role in the GJHQHLRSD-UC network. Through a series of calculations, small molecules of diop, kaempferol, worenine, Palmidin A, and ginsenoside Rg3 ligands were selected. Molecular docking simulations were performed for selected target genes and small molecules. The docking results showed that five targets could directly couple with five bioactive compounds. Moreover, the following displayed strongest combined effects: EGFR with kaempferol, ERK1 with worenine, STAT3 with Palmidin A, BCL2L1 with diop and VEGFA with ginsenoside Rg3 (Figure 7).

## 4. Discussion

UC is a precancerous lesion with lifelong recurrence tendency, which requires long-term medication. Its typical clinical manifestations include abdominal pain, diarrhoea, and purulent stool, among which abdominal pain and frequent defecation severely affect the quality of life of patients with UC [18]. A Chinese study found that the prevalence of anxiety and depression in patients with IBD reached 33.1%, which in turn can aggravate the disease severity [19]. More than 240 genetic risk loci are associated with IBD. However, their effects on the disease are poorly understood [20]. Owing to the complex aetiology and pathogenesis of UC, various modalities are used for its treatment, including the administration of 5-aminosalicylic acid, glucocorticoid, immunosuppressant, and antibiotics, as well as surgery [21–23]. However, drug resistance, drug dependence, and adverse reactions have further limited the clinical effect of pharmacological therapy. Thus, IBD treatment is far from optimal, and currently, the prognosis of patients is not that satisfactory.

Alternative therapies represented by TCM have been reported increasingly in recent years [24–27]. In China, TCM prescriptions based on Han Re Bing Yong Fa have been widely used in UC treatment, with preferable efficacy and safety [28–30]. Basic studies demonstrated that modified BXXXD, a formula similar to GJHQHLRSD, can effectively alleviate UC as well as relieve depression and UC through targeting VEGFA, TNF, STAT3, EGFR, and others [31–33].

However, the scientific explanation of Han Re Bing Yong Fa in treating UC currently remains unclear, which indicates the need for conducting more basic studies to better understand the scientific connotation of the TCM Han Re Bing Yong Fa therapeutic principle. The isolation of artemisinin was inspired by the use of *Artemisia annua* in TCM, which is a typical outcome from the research and mining of TCM theory [34]. Network pharmacology and molecular docking analysis are computed prediction tools offering results that can provide a direction for future research, such as revealing scientific evidence for the TCM principle of Han Re Bing Yong Fa.

The reason TCM treatment of UC has become a research hotspot may be related to its complex pharmacological action featuring the multitarget and multipathway approach. UC pathogenesis is related to pathogenic factors such as abnormal gut microbiota, immune response dysregulation, environmental changes, and gene variants [35]. In this study, the Venn diagram showed that the therapeutic effect of GJHQHLRSD on UC was related to 140 genes (Figure 2). Furthermore, seven target genes were screened by the cluster analysis: *BCL2L1*, *S1PR5*, *ALOX5*, *NR3C1*, *NR1I2*, *CYP2D6*, and *LPAR6*. These target genes are involved in physiological processes such as apoptosis and inflammation as well as hormone and immune regulation. Therefore, these targets might play an important role in the activity of GJHQHLRSD against UC. A network pharmacology study has found that Baitouweng decoction (BTWD) may alleviate UC through multiple targets and pathways [36]. The BTWD has been found to also alleviate inflammation in the mouse model of colitis, which may be related to a variety of signaling pathways, including the modulation of intestinal microflora and inflammatory signaling pathways, such as IL-6/STAT3 [37]. As is known, studying the effect of TCM on human health has always been challenging because of the complex composition of Chinese herbal medicine. The integral and systematic characteristics of the growing field of network pharmacology research into TCM are consistent with TCM's holistic view and principle of syndrome differentiation and treatment. For this reason, some researchers use data mining technology to study TCM. Although the research methods of network pharmacology has some shortcomings, it provides a novel way to study the complex systems of TCM by revealing drugs' regulatory mechanisms through the integration of a large amount of clinical and experimental data and scientific verification [38].

Currently, the primary strategy of IBD is to balance the excessive immune response of the intestinal mucosa so as to restore the epithelial regeneration of colon. Epidermal growth factor is an activated ligand of EGFR, which can alleviate disease by directly targeting intestinal mucosal healing. EGFR activation therapy works well in clinical practice but has not shown progress in the past few decades, partly because its long-term use may cause cancer. Animal studies have shown that early administration of gefitinib, an EGFR kinase inhibitor, can increase the tumour size, whereas its late administration can reduce the tumour size. EGFR plays an important role in the pathological development of IBD, especially CAC [39, 40]. The mechanism of EGFR in IBD treatment is unclear, yet most studies show that EGFR is closely related to cytokines and mitochondrial autophagy [41, 42]. Previous studies found that A disintegrin and metalloproteinase-17 and EGFR can alleviate UC by reliving inflammation and restoring intestinal barrier [43, 44]. EGFR activation promotes cellular proliferation, differentiation, survival, and wound healing in several cell types [45]. Moreover, the specificity of UC is still associated with an altered EGFR expression, and the rate of epithelial apoptosis and proliferation is determined by the histological activity of inflammation [46]. The PPI network analysis demonstrated that seven target genes of GJHQHLRSD were related to cell proliferation, apoptosis, and immune regulation (Figure 4), which is accordance with the principle of balancing excessive immune response in UC treatment.

In addition to recent research on EGFR and excessive immune response in UC treatment, research on mitochondrial autophagy demands scientific attention. Because epithelial barrier repair in colitis is dependent on energy, EGFR tyrosine kinase inhibitors and mitochondrial autophagy regulation are particularly important. Xianglian pill reduced DSS-induced acute colitis in mice by inhibiting the secretion of proinflammatory cytokines and enhancing autophagy [47]. Moreover, a study on compound Sophorae decoction found that TCM can inhibit UC-associated carcinogenesis by fighting inflammation and regulating apoptosis and mitochondrial autophagy [48], which suggest that mitochondrial dysfunction is critical in UC-associated carcinogenesis [49]. In light of these findings, mitochondria may become a new pharmacological target for the prevention and treatment of IBD [50, 51]. This speculation is consistent with the results of this study. The KEGG and GO enrichment analyses results indicated that GJHQHLRSD functions are regulating the EGFR signaling pathway in UC treatment (Figure 8). In this study, other effective biological processes involved in UC treatment included cancer-related as well as inflammation and viral infection signaling pathways, such as the “MicroRNAs in cancer,” “TNF signaling pathway,” and “JAK-STAT signaling pathway.” Growing evidence demonstrates that microRNA-mediated posttranscriptional regulation is important in autophagy in IBD [52]. MicroRNA was found to be involved in regulating the occurrence and development of UC in four ways by affecting the intestinal epithelial cell barrier, regulating immune cells, regulating intestinal microbiota, and participating in tumour formation [53]. Baicalin, the active component of Radix Scutellariae, was found to play an antitumour role by regulating dozens of microRNAs [54]. Previous studies on Radix Scutellariae and Coptidis Rhizoma also found that the mechanism of alleviating UC is related to TNF-*α*, STAT3, and JAK-STAT signaling pathways [47, 55–57]. In conclusion, EGFR tyrosine kinase inhibitor and mitochondrial autophagy are key factors in the pathological progression and recovery of UC.

In this network pharmacological study, 71 potentially bioactive compounds of GJHQHLRSD were identified, including kaempferol, worenine, Palmidin A, diop, and ginsenoside Rg3. Kaempferol, present in Ginseng Radix et Rhizoma and Radix Scutellariae, exerts anti-inflammatory and antitumour effects by inhibiting inflammatory factors [58]. Worenine is a major active component of Coptidis Rhizoma, which inhibits colorectal cancer cell growth by negatively regulating HIF-1*α* [59]. Moreover, the molecular docking results revealed that the five abovementioned major compounds of GJHQHLRSD had a high binding affinity to the EGFR in the tyrosine kinase inhibitor signaling pathway (Figure 7). In particular, EGFR with kaempferol and ERK1 with worenine displayed the strongest combined effects. Kaempferol and worenine have definite anti-inflammatory and antitumour effects, consistent with the fact that UC is an inflammation-based precancerous lesion. Collectively, this network analysis suggested that the major active components of GJHQHLRSD work effectively on UC by counteracting inflammation and regulating the EGFR signaling pathway along with other biological processes.

### 4.1. Study Limitations

This study has some limitations. The pharmacological mechanisms of GJHQHLRSD in treating UC were investigated in this study. However, further animal experiments are warranted to ensure the reliability and rationality of the predicted results. In addition, further studies on related mechanisms are required to determine the function of upstream and downstream proteins regulated by key genes. Moreover, key proteins and KEGG signaling pathways must be verified through a scientific experimental design. As GJHQHLRSD is a compound ingredient, further studies are required to scientifically screen its active ingredients, improve OB, and identify adverse reactions.

## 5. Conclusions

The application of the TCM Han Re Bing Yong Fa therapeutic principle has shown some advantages in UC treatment, especially in improving the intestinal barrier function and delaying cancer development. In this study, network pharmacological analysis revealed the characteristics of the action mechanism through which GJHQHLRSD treats UC, which may involve multiple components, targets, and multiple pathways. On the basis of the network pharmacology analysis, GJHQHLRSD achieves anti-inflammatory effects by regulating 141 pathways, included inflammation as well as cancer-related and viral infection signaling pathways, such as the “EGFR signaling pathway,” “MicroRNAs in cancer,” “TNF signaling pathway,” and “JAK-STAT signaling pathway.” Although these pathways have been shown to be strongly associated with UC, some pathways have not yet been shown to be regulated by GJHQHLRSD. Therefore, further studies on related mechanisms are required, especially on the role of upstream and downstream proteins regulated by key genes.

## Figures and Tables

**Figure 1:** Flowchart of UC treatment using GJHQHLRSD based on the network pharmacology approach.

**Figure 2:** (a) Venn diagram of the GJHQHLRSD targets. (b) Venn diagram showing the overlapping target genes between GJHQHLRSD and UC.

**Figure 3:** Network diagram of interaction between the drug component and the target disease.

**Figure 4:** Protein-protein interaction network clusters of common targets for both GJHQHLRSD and UC. (a–g) Clusters 1–6 found using MCODE and had densely connected regions. (h) Comparison of the MCODE scores of different clusters.

**Figure 5:** GO enrichment analysis. (a) Go enrichment analysis of three processes. (b) The BP 20 bubble diagram. (c–e) BP-related gene signaling pathway network.

**Figure 6:** KEGG enrichment analysis. (a) Bubble diagram of the KEGG enrichment analysis. (b) Gene distribution of the EGFR signaling pathway. (c) GJHQHLRSD against the UC target-pathway network.

**Figure 7:** (a) Binding energy scores of molecular docking. (b−f) Binding modes of target genes and ligand proteins.

**Figure 8:** EGFR signaling pathway of GJHQHLRSD against UC.

## Data Availability

The figures used to support the findings of this study are included within the article, and the data used to support the results are available from the corresponding author upon request.
